# The Big Data Model for Urban Road Land Use Planning Is Based on a Neural Network Algorithm

**DOI:** 10.1155/2022/2727512

**Published:** 2022-09-13

**Authors:** Sunan Tu, Ming Zhang

**Affiliations:** ^1^School of Architecture, Southeast University, Jiangsu, Nanjing 210096, China; ^2^Keltai Real Estate Development (Nanjing) Co., Ltd., Jiangsu, Nanjing 210005, China

## Abstract

The spatial differentiation of land use induces traffic demand and guides the construction of traffic supply; traffic conditions are an important influencing factor in determining the nature of land use, and there is a close interaction between the two. This study uses a neural network-based approach at the urban grid level to portray representative phenomena of urban development and analyze the interaction between transportation and land use. The results reflect the model's effective simulation of urban laws, and the case study reveals the differences in the laws of different cities, to guide the benign development of cities and transportation. This article firstly conducts a study on the theoretical foundation; compares the development history, planning, and design methods and practical experience of road planning and resilient planning; summarizes the experience of resilient road system design; and analyzes the future development trend, based on the above basic theoretical research, to develop research ideas and methods. Secondly, the scenario analysis method is explicitly applied to analyze various scenarios that may occur in the future development process of simulated urban roads and rank the scenarios based on the probability of occurrence. For the impact of traffic on land use, the concepts of vitality and potential are introduced, and a multidimensional long and short-term memory network (MDLSTM) model is established. The model takes into account land use lags and potential transfer and has relatively higher prediction accuracy. The results show that larger cities with urban dominant industries and tertiary industries also have higher land use potential and the more significantly influenced by traffic.

## 1. Introduction

Transportation activities are an important part of modern urban life, and transportation facilities are the yardstick and link to economic and social development and urban growth. With accelerated urbanization, the problem of urban traffic congestion has become increasingly serious. The spatial distribution of land use generates transportation demand, and location and transportation conditions are important influencing factors of urban land differentiation, and modeling and quantifying the mutual influence process between them has been a key topic in the field of sustainable urban development [1]. From a macroscopic point of view, the evolution of urban development is always accompanied by changes in land transactions and transportation patterns. The high concentration of residential neighborhoods and the separation of jobs and residences have profoundly affected the spatial distribution patterns of traffic in many large cities at present, and the monocentric and borderless spatial structure of some cities has led to an unstoppable slide toward long-distance, high-frequency commuting, and car-led traffic patterns. Urban transportation and land use have a close coupling relationship. In the short term, the spatial distribution of urban land use is relatively static, and various areas with different land-use properties complete the exchange of people and products through urban transportation links, that is, urban land use patterns determine the generation and spatial distribution of urban transportation [2]. In the long term, the construction of transportation infrastructure and the supply of transportation services improve accessibility, and the increased commuting costs of traffic congestion reduce the land value of the area, and this difference in value further adjusts the land development process through the individual choice behavior of urban residents, thus affecting the urban spatial structure [3]. The macroscopic relationship between these has been systematically studied by a series of more mature theories such as accessibility theory, transportation planning theory, and transportation supply-demand balance theory from a general perspective.

The complexity of urban laws and influencing factors also pose a challenge for the identification of traffic and land use integration laws. Cities have a large number of nonlinear, multi-factor simultaneous effects and other complex development and change laws. In parts of time, there is often a lag in the construction of various types of facilities in cities; land use types do not respond in real-time to make changes after traffic conditions change, and it takes time to plan and build transportation facilities after land-use types change, which objectively affects the accuracy of data-driven models [4]. Spatially, different regions, spatial units, land use types, and influencing factors within the city have different spatial interactions, and the spatial correlation of land use and traffic demand is often significantly correlated with distance, while the spatial correlation of traffic supply is directional and often distributed along the road network, bus network, or rail network, which makes it similar to meta-cellular automata, convolutional. This makes it difficult to accurately simulate models like beta cellular automata, convolutional neural networks, and other models with “translation-invariant” properties. In terms of influencing factors, the number or size of most commercial facilities reflects the demand of urban residents for this type of urban service, but in terms of facility quality, the demand for high-level facilities is not easily reflected by static indicators such as floor area and floor area ratio. In this article, we use convolutional neural network-multidimensional long and short-term memory network (CNN-MDLSTM) to fit the basic attributes of the network, road network density, and various types of land use property scores of the parcel as the input and traffic generation attraction as the output, and the prediction accuracy of traffic generation attraction and the influence of various types of land use and indicators are analyzed. The factors of the prediction accuracy of traffic attraction and the influence of each type of land use and each index on the prediction accuracy of traffic attraction were analyzed. Finally, we used the convolutional neural network and cross-long and short-term memory network (CNN-CLSTM) to fit the basic attributes of the network, the scores of various land-use properties and traffic attraction as input, and the road network density, the total number of surrounding bus stops, and traffic facilities as output and analyzed the relative influence of each index on the output.

## 2. Related Work

The complexity of urban laws and influencing factors also pose a challenge for the identification of traffic and land use integration laws. Cities have a large number of nonlinear, multi-factor simultaneous effects, and other complex development and change laws. In terms of time, there is often a lag in the construction of various facilities in cities; land use types do not respond in real-time to make changes after traffic conditions change; and it takes time to plan and build transportation facilities after land-use types change, which objectively affects the accuracy of data-driven models.

Some scholars have preliminarily studied the theory of intensive land use, put forward the relevant concepts and connotations of intensive land use, and determined the basic contents of intensive land use. Jun [5] put forward reasonable improvement methods from urban land use structure and layout to promote coordinated and sustainable urban development. Qi et al. [6] considered the connotation of land-intensive utilization from three different perspectives, such as the perspective of matching the scale of urban development and the scale of industrial structure, the perspective of the structure and reasonable distribution of the functions of each land use in the city, and the perspective of the input-output requirements of each land use. From different levels of the literature, [7] argues that different cities present different urban conflicts and characteristics, and need to combine different urban development levels and positioning, and puts forward intra-city land rectification programs and measures. Mu et al. [8] construct and evaluate land-use efficiency evaluation systems from macroscopic to microscopic perspectives for commercial, industrial, and residential land use types in municipal districts. Wu et al. [9] propose that the land type of urban low-utility land is urban construction land first, and on this basis, urban low-utility land can be judged by two indicators: building capacity and land output efficiency. Some government departments not only consider the level of land use and input-output efficiency, but also consider whether urban land is low-utility land in terms of land layout, level of supporting facilities, and ecological and environmental protection. The article [10] evaluates the efficiency of industrial land use in terms of land use output and social services based on the micro-plot scale and explores the relationship between land use structure and its efficiency. The literature [11] studied the effect of far-left-turn traffic implementation at signalized intersections and proposed a microscopic traffic model applicable to typical urban areas, and evaluated the left-turn organization of different signal-controlled intersections. The literature [12] described the operation law of mixed traffic flow at signalized intersections by establishing a microscopic traffic simulation model and studied the before-and-after effect of left-turn traffic flow, left-turn vehicle ratio, and dedicated lane length based on the waiting time of vehicles after the stop line. Chen et al. [13] used detectors to collect left-turn traffic flow and delay under various types of phases with constant periods and phases.

The data relating to the errors and the relationship model between the flow and delays were established. The literature [14] investigated the conditions for setting left-turn lanes and their application in practice proposed that left-turn lanes can effectively organize the left-turn traffic flow at planar intersections, and evaluated the safety and efficiency of left-turn lanes. Chen et al. [15] emphasize that the road network form and streets should become an important public space reorganization linked to the urban design level in the design optimization of the slow walking system, while the spatial forms of streets and road networks are closely related to other spatial design contents and deep social, economic, and environmental contexts. Saralioglu and Gungor [16] studied the development process of the green transportation concept and proposed that, firstly, the construction of horizons on the human sightline should be considered from the scale of people themselves. Secondly, it is necessary to create a traffic information platform using cell phone terminal data. Finally, it is proposed that effective measures should be taken to improve the competitiveness of urban public transportation.

## 3. Optimization Algorithm of Urban Road Land Use Planning Based on a Neural Network Algorithm

### 3.1. BP Neural Network Land Allocation Optimization Algorithm Based on Entropy Power Method

Since this article needs to quickly identify low-utility sites in cities for further screening by subsequent planners based on actual conditions and further determination of urban renewal timing and renewal strategies, reducing human subjective involvement is the main way to improve the low-utility site identification process. The complex evolution mechanism of geographic scenes determines that giving physical meanings to indicators requires the introduction of machine learning algorithms with autonomous learning capability and self-adaptive ability, which can be used to mine the data and learn the intrinsic complex connections behind the data, to calculate the indicator weights based on the geographic meanings. Therefore, this article adopts the method of combining the entropy method and machine learning algorithm to objectively reflect the importance of index attribute information in the whole evaluation system by entropy method and then combines with machine learning to correct the weights determined by the entropy method [17]. The entropy weight method is an objective method of calculating weights evolved from the discipline field of the signal system, which is developed by measuring the amount of information in the system, called information entropy, and the higher the information entropy in the system, the more orderly the system represents; on the contrary, the more chaotic the system is. For the evaluation system, the information size of the evaluation index also represents the degree of the orderliness of the system. Spatially, different regions, different spatial units, different land use types, and different influencing factors within the city have different spatial interactions, and the spatial correlation between land use and transportation demand is often significantly correlated with distance. The higher the information size of the evaluation index, the higher the information entropy, which indirectly represents that the index occupies an important position in the system.

The indicator weights determined by the entropy weight method depend on how much attribute information the indicators contain among all indicators, and their weight values rely heavily on the sample data, lacking horizontal comparison among indicators, resulting in the indicator weights contradicting the importance of the actual impact on land-use efficiency, and finally obtaining unreliable low-utility land identification results. Land use is a complex system, and the assessment of land-use efficiency is also a complex nonlinear process. To accurately assess the land-use efficiency situation and identify low-utility land, the learning mechanism of indicator weights should be designed based on the complex system, and the systematic characteristics of the indicator factors should be explored. In this article, the initial weights of evaluation indicators obtained by the entropy weight method are used as input data, and the learning mechanism of the BP neural network is used to reverse calculate the node values of each node in the output layer and the implied layer as well as the corrected amount of node weights, and the neural network is used to identify the unknown connections among indicators and the positive knowledge inference to correct the weights obtained by entropy weight method and reduce the deviation of the weights obtained based on the pure information confusion so that the weights are closer to the actual situation [18]. Based on the initial weights of indicators obtained initially by the entropy weighting method, the land inefficiency identification index is calculated and normalized with the initial land inefficiency identification index as the learning sample, that is, the input layer, which is represented by the matrix as

(1) $$\begin{array}{c} A_{mn}=\left(\begin{array}{ccccc} a_{11} & ... & a_{1k} & ... & a_{1n}\\ ... & ... & ... & ... & ...\\ a_{i1} & ... & a_{ik} & ... & a_{in}\\ ... & ... & ... & ... & ...\\ a_{m1} & ... & a_{mk} & ... & a_{mn} \end{array}\right). \end{array}$$

Denote the desired weight by *w*, the number of nodes in the hidden layer by *p*(*x*), and the number of nodes in the hidden layer by *δ*, where

(2) $$\begin{array}{c} w=\frac{kx+\delta }{p^{2}\left(x\right)}+Cp\left(x\right). \end{array}$$

The vector of weights of the connections between the nodes in the implied layer and the output layer is denoted by (*x*), where *k* denotes the connection weight of the *k*th node. The output layer is the weight of each indicator with a vector $\overset{⟶}{O}\left(x\right)$, with V denoting the connection weight between the input layer and the implied layer, indicating the connection tightness between the nodes. The transfer function is selected as the Sigmoid function to train the samples.

(3) $$\begin{array}{c} G\left(x\right)=V\int^{}\left[kx^{2}+p\left(x\right)\right]dx+\overset{⟶}{O}\left(x\right). \end{array}$$

The specific process and basic steps of the road land weight correction model using the BP neural network in this article are shown in Figure 1.

The network error for each sample during training and the total cumulative network error is calculated as

(4) $$\begin{array}{c} {\text{g}}_{k}=T\left[f_{k}\right]=\overset{k}{\underset{i=0}{\sum }}P\cdot f_{i}. \end{array}$$

The model is generally divided into three layers of structure: an input layer, an output layer, and an implicit layer, where the input layer is the initial value of internal and external indices and index standardization obtained by using the initial weights, and the output layer is the initial weight of entropy weight method. For the two types of land use, the indicators of internal properties and external characteristics need to be optimized separately, so four times neural network weight optimization is carried out according to the model structure, that is, the six indicator values and the initial index of internal properties of road use are used as the input layer nodes after standardization of internal properties of road use, and the weights of indicators of internal properties of road use are used as the output layer; the seven indicator values and the initial weights of external characteristics of road use after standardization of external characteristics of road use are used. In the same way, the same training is carried out for all industrial land parcels. In the BP neural network algorithm, the *S*-type function is generally used to ensure that the activation function is derivable everywhere. The logistic function is suitable for the activation function required to calculate the weights in this article because the output values of the training samples are the weights between 0 and 1, and all the values are guaranteed to be in the interval [0, 1] compared with the general linear function.

### 3.2. Urban Road Land System Planning Scheme

The establishment of the evaluation index system of the new area road network system requires the selection of suitable evaluation indexes from the technical evaluation indexes of the road network. The evaluation of technical indicators can be done from several aspects such as construction level, the geometric topology of the road network, and connection quality [19]. However, without a large-scale traffic survey, many evaluations may not be analyzed due to the lack of data for the current situation of a new city with almost no traffic demand. Therefore, in this article, the technical indicators of the road network are divided into four levels: road characteristics, access depth, service characteristics, and traffic characteristics, some of which may reflect two or more levels at the same time and there are some duplications. Road characteristics reflect the nature of the planned road function and construction level in the case of clear road traffic planning.

Under can be described from the perspective of road network technical level, per capita road area, road network density, arterial road network density, road network connectivity, road network capacity, and pavement paving rate. For new urban areas generally in the construction process, there is the problem of pavement rate road network is completed and there is no problem of poor pavement rate. Access depth reflects the connectivity and convenience of the road network. In the case of clear traffic demand and planning, road network can be described from the perspective of road network density, road network connectivity, connectivity index, road network accessibility, road network nonlinear coefficient, unit traffic accessibility, unit traffic nonlinear coefficient, etc.

The method of integration degree uses spatial syntax indicators and models to study the spatial morphology of road networks to find the interaction between the spatial morphology of road networks and urban spatial morphology. Integrating the pulse of Changsha's urban growth with the fitting of cab big data, it is proved that the method of aggregation degree can be used to reflect the spatial morphology of the road network and analyze its relationship with the urban spatial morphology [20]. The indicator weights determined by the entropy weight method depend on how much attribute information the indicators contain among all indicators, and their weight values rely heavily on the sample data, lacking horizontal comparison among indicators, resulting in the indicator weights contradicting the importance of the actual impact on land-use efficiency, and finally obtaining unreliable low-utility land identification results. The spatial sentence method integration index can be used at the general planning level to identify the central tunnels, districts, and box shot axes, provide traffic and morphological basis for general planning zoning, and provide data support for zoning differentiation requirements; at the control planning level, it is mainly used to identify roads with high integration degree, check and optimize the layout of convenient land, and check and optimize the number of road lanes, rail lines, and conventional bus lines; at the revision planning level, it is mainly used to identify roads with high integration, find the preferred path for encrypting the branch road network, and optimize the integration and layout of related buildings, supporting facilities and sites in the project. The “system quantification” assessment can be used to comprehensively assess the supply of the road network carrying capacity (also includes the comprehensive traffic carrying capacity of the road network as a carrier), the traffic demand, and traffic patterns corresponding to the land-use planning, of which the grid method is the supply-side assessment, compared with the previous single-density assessment, there are more density indicators, and indicators reflecting non-homogeneity. The integration degree method reveals the non-homogeneity of the road network in a more systematic way. The saturation method directly assesses the supply and demand, which is the key to recognizing and predicting the traffic supply and demand corresponding to the planning and to plan the traffic supply and demand balance.

Among them, road network density is an important indicator of the quality of urban traffic road network layout can reflect the number and level of urban road network construction reflects the quality of urban road network layout. Service characteristics reflect the road users according to the traffic state from the speed, comfort, convenience, economy, safety, and other aspects of the degree of service received. In the case of clear road traffic planning and road, traffic flow can be described from the perspective of road network service level, road network ratio, and road network load degree uniformity. Among them, the level of service reflects the level of quality of operational services provided under certain traffic conditions road network load uniformity reflects the degree of difference in congestion on each route in the region. Traffic characteristics reflect the performance of traffic flow on the planned road. Based on a clear section of traffic demand, it can be described from the perspective of road network traffic speed, road network traffic density, and road network flow [21]. Among them, road network traffic speed includes simple average traffic speed, flow or distance weighted average traffic speed, and flow distance weighted average traffic speed. It is assumed that accurate prediction of traffic demand and clear road network planning follow the principle of indicators as few as possible and indicators all quantitative. This article extracts 15 indicators from 4 levels of road characteristics, access depth, service characteristics, and traffic characteristics to establish a three-tier indicator system. These indicators can reflect the essential characteristics of the road network to achieve our goal of road optimization. The structure of the evaluation index system of the new area road network system planning scheme is shown in Figure 2. The definition of each indicator in this evaluation system is consistent with the model in the conventional technical evaluation.

Due to the different scales used for each technical indicator, it is necessary to standardize the indicators to calculate the selected indicators. Here, the linear extremum method is used to establish the affiliation function to normalize each indicator. The expressions are as follows for the larger and better indicators.

(5) $$\begin{array}{c} H\left(x\right)={\sum^{}}_{i-1}^{n}p_{i}\ln\frac{1}{p_{i}}. \end{array}$$

The consistency ratio of the judgment matrix can be obtained by the above method and then determine whether it passes the consistency test. The weight coefficients that pass the test can be used as the weights of each index. In the process of moving from the current situation to the future, various spatial and temporal scales of planning and self-organization come into play at the same time. Generally speaking, the long-term planning, the larger the spatial scale considered, the more it favors the structural order, and the more recent planning, the more it needs to be detailed and precise and operable, and the more it favors the functional order. Structure and function are two sides of the same coin for a specific space, and any construction behavior and planning can find its corresponding spatio-temporal scale and target, and make corresponding macro and micro, near and long-term integration [22]. From the point of view of planning regulation, the larger the spatio-temporal scale is, the larger the planning is in the knotty framework, only the objectives need to be specified for the lower level planning, thus the structural framework and the objectives of the lower level are its focus and the focus of planning assessment, the indicators of structural elements and the spatial layout and implement are the elements to be assessed. Planning at smaller spatial and temporal scales, within the framework of upper level planning, also needs to fully correlate macro-structure and context with relevant details to better play the role of self-organization and better realize spatial functions.

## 4. Dynamic Balance of Urban Road Land-Use Planning Based on a Neural Network Algorithm

The goal of urban road network planning is to provide a planning blueprint and construction basis for achieving a balance between traffic supply and demand, and the corresponding assessment is whether a balance between traffic supply and demand can be achieved, and the whole process of planning should be a process to achieve a dynamic balance. From the research of the current situation, the formulation of the planning scheme to the decision-making, implementation, feedback, and even adjustment of the planning scheme, a set of scientific and reasonable evaluation methods are needed to assess the current situation, the rationality of the planning scheme, and the adaptability of the plan after implementation. From the perspective of demand management, land-use planning should interact with road traffic planning and match each other to ensure land for road traffic and realize its traffic carrying capacity, but also scientifically plan the nature and intensity of land parcels and rationally plan traffic demand. Therefore, the introduction of evaluation in the planning process is the need to improve the planning process, and the planning evaluation flow chart is proposed by drawing on the neural network algorithm of complex systems, as is shown in Figure 3.

In physical planning, the object of planning is mainly physical space, focusing on the study and arrangement of block land space of various natures and network road space made up of a combination of linear space, and there is an interactive relationship between road network planning and the land planning of the areas it serves. From the perspective of traffic supply and demand, the land planning of other spaces corresponds to the corresponding traffic demand, the amount of traffic demand and spatial distribution is due to the nature of the land and intensity of other spaces layout triggered by the supply of the road network that the road network carrying capacity for (including motor vehicle traffic carrying capacity for, dependent on the road network of rail transit and The balance between the volume and spatial distribution of demand (including motor traffic carrying capacity, rail and conventional bus carrying capacity attached to the road network, and slow traffic carrying capacity) depends on the balance of planned land supply. The assessment of the dynamic balance of traffic supply and demand through the above process contributes to the preparation of urban planning and its implementation.

From the viewpoint of supply carrying capacity, the self-organization of adaptive subjects and their elasticity of multi-modal combination of travel provide the basis for the dynamic balance of urban traffic, and the road network planning at all levels of statutory planning should provide a framework for self-organization and provide target requirements and spatial guidance for the planning of public transport line network, especially the rail line network among them. From the point of view of demand management, land-use planning should interact with road traffic planning, matching each other, not only to ensure that road traffic land achieves its traffic carrying capacity, but also scientific planning of land parcel land nature and intensity and rational planning of traffic demand. From the point of view of urban form, the road network form as a whole should match the urban spatial form. From the same circle theory, the city is also a district, and box shot axis integration is high, good economic benefits, traffic demand, should be more bearing capacity supply [23]. The middle is the area often the land price highland, the proportion of road occupation is not likely to be too high, the difficulty of building higher grade roads, and thus the need for a much higher proportion of public transport sharing than other areas, the need for road space in as much as possible to plan the rail and other public transport facilities.

From the perspective of complex adaptive system theory, the node is a space enclosed by its surrounding road network dividing other spaces, and its size and shape are directly influenced by the density and shape of the road network. Completeness is a measure of the success of a retrieval system in detecting relevant results from a sample set, that is, the ratio of relevant results detected to the total number of objects in the retrieval system; accuracy is a measure of the signal-to-noise ratio of a retrieval system. The nature of the land and volume ratio of the node space determines the demand and characteristics of the road traffic of the “main body,” that is, the “traffic flow.” The relationship between the road and the public transport capacity it carries and the “traffic flow” affects the utilization of the road and thus the utilization of the node space. The grid method uses the method of comparing standard indicators to assess the size, car-carrying capacity, and shape of the road network as a physical network, derives the standard indicator system and general intersection spacing, proposes a statistical calculation table to facilitate the comparison of indicators, and then draws conclusions from the table calculation and intersection spacing comparison. The grid method is based on the norms and experience of the road supply perspective assessment method, and also needs to cooperate with other methods of assessment. From the research progress of the national standard, the urban morphology has an increasingly influential role in road network planning, and the non-homogeneity of urban space indicates that the national standard index cannot guide the control plan of all lots, much less the node revision plan.

A comprehensive and systematic comparison with an index system based on the needs of each level of planning is the basis for evaluation, and more empirical research is needed in various places to accumulate experience and data. The saturation method uses traffic indicators and traffic models to analyze the relationship between traffic demand and supply and proposes an overall saturation table to grasp the relationship between traffic supply and demand in the statutory urban planning stage, while the “four-stage” traffic model can output the saturation of each road section, which is a visual reflection of the traffic supply and demand in the future years under the implementation of the plan [24]. In the general plan, the overall saturation table mainly calculates and grasps the average saturation of the backbone road network, while constructing as detailed a traffic model as possible to grasp the saturation forecast of each road as accurately as possible. In the revision and road planning and design, the evaluation results from the master plan and control plan preparation and decision-making are used to analyze the system connection between the project and the lot and the city, and to improve the design level and project value.

## 5. Experimental Verification and Conclusion

### 5.1. Algorithm Parameter Testing

After screening, the main parameters selected for the algorithm include the sampling window size is 9, the evaluation region size is 3, the number of convolutional kernels is 4, the convolutional kernel edge length k*d* = 7, the data segment length is 1500, the optimizer is RMSProp, the learning rate is moving average exponential decay mode, and the segmentation mode is “window-to-window” mode with high model prediction accuracy and training speed. In the long term, the construction of transportation infrastructure and the supply of transportation services improved accessibility, and the increased commuting costs of traffic congestion reduce the value of regional land use. The model hyperparameters to be further validated are the number of neurons in the hidden layer of the cross-long-short memory network and the orbit-long-short memory network. In the cross-long-short memory network, the number of hidden layer neurons from 1 to 20 was tested considering the model training time reason. As shown in Figure 4, for each value of the number of hidden neurons, 100 cycles of training were performed, the percentage error of the test set was collected, and the trough of each 100 values corresponded to the highest value of the test accuracy, and it was found that the model with 11 hidden neurons had better results.

The number of hidden layer neurons from 1 to 20 was tested in the railroad long and short memory network, and each peak shows the training process when the test accuracy reaches its highest point, and the model with 7 hidden layer neurons was found to have better prediction results. The CNN-CLSTM model was compared with various neural network models including feedforward neural networks (FFNN), convolutional neural networks (CNN), and multidimensional long and short-term neural networks (MDLSTM) in terms of training speed and model effectiveness. In addition to the constituent models, feedforward neural networks were also used as control models for the comparison of model effects due to their simple model structure. The training speed was reflected by the performance of each model on the training set, and the model effects were evaluated by the performance of individual models on the test set. About 100 steps of training were performed for each model, and the percentage errors of the training and test set data are shown in Figure 5.

From the percentage error results of the training set, it can be seen that the CNN-MDLSTM has a relatively fast convergence speed among all models within 30 training steps, and the improved CNN-MDLSTM model converges faster than other models after 30 training steps. From the prediction effect, the improved CNN-MDLSTM significantly improves the accuracy of the results. Adding the directional prior information reduces the prediction model error from 16.36% to 13.30%, with an accuracy improvement of about 3%; adding the rail traffic prior information reduces the error from 16.32% to 13.30%, with an accuracy improvement of about 3%.

### 5.2. Evaluation Index Weight Optimization Example Validation

Completeness rate and accuracy rate are important metrics commonly used in the field of information retrieval to reflect the effectiveness of retrieval. Completeness rate is a measure of the success of a retrieval system in detecting relevant results from a sample set, that is, the ratio of relevant results detected to the total number of objects in the retrieval system; accuracy rate is a measure of the signal-to-noise ratio of a retrieval system, that is, the percentage of correct results detected to the total number of results detected. As shown in Figure 6, the detection rate and accuracy rate of residential land use are 57.14% and 85.71%, respectively, and the detection rate and accuracy rate of road use are 67.35% and 86.84%, respectively, with the accuracy rate reaching more than 80%, but the detection rate is low, indicating that the low-utility land evaluation and identification method proposed in this article can identify the low-utility land within the city more accurately, and some errors in some of the identification levels and a very small percentage of them are not identified, but the overall identification is good. Land-use types do not respond in real-time to make changes after traffic conditions change, and it takes time to plan and build transportation facilities after land-use types change, which objectively affects the accuracy of data-driven models. The main goal of this article is to first identify the parcels that may belong to low-utility land as much as possible, and then the staff will conduct field research on the specific parcels to determine whether they are classified as urban renewal objects, thus reducing the research workload and therefore focusing more on the accuracy rate, which leads to some parcels being classified below the moderate level.

In this article, taking the road land type as an example, the optimized weights were calculated for 186 road land parcels, and the internal property index and external characteristic index of the road land were calculated by weighting the initially determined weights, and the standardized internal and external initial index values and the internal and external indices were used as the input nodes of the BP neural network, respectively, and the initial weights were used as the output nodes to obtain the corrected values of the weight of each index in the land type. The results are shown in Figure 7.

As can be seen from Figure 7, the initial values of the normalized internal and external indicators of the road land and the internal and external indices are used as input to the initial weights for the BP neural network model correction, and the overall operational accuracy *R* values reach 0.9942 and 0.97882, respectively, and the training learning accuracy is good, which can realize the mining of the data features between the internal indicators based on the existing objectively determined weights, and the learning training process In the process of learning and training, the weights are adjusted, and the weights before and after the final adjustment are good. As can be seen from the figure, the optimization error (Error) of the internal property and external feature indicators of road land is much smaller than the set target error of 0.001, and the training results are good. The adjusted weights of the internal property indexes of the BP neural network are 0.1411, 0.1464, 0.2012, 0.2037, 0.1536, and 0.1540, and the initial weights obtained by the entropy weighting method can be seen, to reduce the weight of the building layer index in all the indicators, increasing the weight of the building density and building age indicators, and the weight of the site property and The adjusted weights of external characteristics of the BP neural network are 0.1067, 0.1911, 0.1241, 0.1086, 0.1149, 0.1635, 0.0476, and 0.1435 in order. Neural network modified weights, the weights of the infrastructure completeness index are more prominent. It can be seen that the index weights modified by the BP neural network algorithm retain the original meaning of the entropy weight method and also make the index weights more objective, so the weight modification method based on BP neural network can be applied in the evaluation of land-use efficiency.

Low-utility land is identified for all road land type parcels in a district, and the overall distribution is shown in Figure 8 after the division according to the low-utility evaluation grade. From the figure, it can be seen that the heavy low-utility land in the district is mainly distributed in the northeast corner of the district, and the heavier low-utility land is mainly distributed in the northeast and south areas, and the land-use situation of the whole district is mainly lighter low-utility grade and medium low-utility grade, and the overall land-use efficiency situation is good.

Through statistical analysis of the obtained results, there were 38 low-utility land parcels with moderately low-efficiency grade or above, accounting for 20.32% of the total number of road land parcels, including 8 heavy low-utility parcels, 30 heavier low-utility parcels, 56 moderately low-utility and lighter low-utility parcels each, and 37 light low-utility parcels, with the grade above moderately low-utility being the focus of this article. This article randomly selects the streetscape data of parcels with heavy inefficiency grades and heavier inefficiency grades in the study area for viewing and verification and finds that the overall identification effect is good using the low-utility land identification and evaluation method proposed in this article, and can accurately identify parcels with serious inefficiency in land use. From the overall spatial distribution, the inefficient road land above the medium level shows a more obvious clustering feature and a circling structure decreasing from the center of the area to the outer edge step by step.

## 6. Conclusion

This article compares the concept and characteristics of the urban central area and low-utility land in the central area, discusses the formation mechanism and influencing factors of low-utility land in the urban central area, and designs a big data model for urban road land planning. The concept and criteria for defining low-utility land in urban central areas are determined, and land-use data, road data, river and water system data, service POI data, statistical yearbook data, and other auxiliary data are selected as basic data. The grid method uses the method of comparing standard indicators to assess the size, small car-carrying capacity, and morphology of the road network as a physical network, derives the standard indicator system and general intersection spacing, proposes a statistical calculation table that is convenient for comparing indicators, and then draws assessment conclusions by comparing the table calculation and intersection spacing. Finally, the feasibility of the proposed index system and the index weight determination model is verified by the case study.

## Figures and Tables

**Figure 1:** Flow chart of weight correction model based on BP neural network.

**Figure 2:** Evaluation index system of road network planning scheme in the new area.

**Figure 3:** Framework diagram of dynamic planning of urban road land based on a neural network algorithm.

**Figure 4:** Percentage error of the model corresponding to different number of neurons in the hidden layer of the crossover neural network.

**Figure 5:** Percentage error of training set for each model.

**Figure 6:** The search completion rate and accuracy rate of different site types.

**Figure 7:** Road land-use internal property index weighting correction.

**Figure 8:** Distribution of evaluation results for identification of low-utility land for road use.

## Data Availability

The data used to support the findings of this study are included within the article.
